# Prediction of Gestational Diabetes Mellitus under Cascade and Ensemble Learning Algorithm

**DOI:** 10.1155/2022/3212738

**Published:** 2022-07-14

**Authors:** Jie Zhang, Fang Wang

**Affiliations:** ^1^Department of Obstetrics, Xianyang Central Hospital, Xianyang City 712000, China; ^2^Department of Hematology Endocrinology, Xianyang Hospital of Yan'an University, Xianyang City 712000, China

## Abstract

Gestational diabetes mellitus (GDM) is one of the risk factors for fetal dysplasia and maternal pregnancy difficulties. Therefore, the prediction of the risk of GDM in advance has become a big demand for millions of families. Therefore, machine learning technology is adopted to study GDM prediction. Firstly, the data is preprocessed, and the mean value is used for outlier processing. After preprocessing of the data, the IV value method is used to screen the features. Of the 83 features in the original sample data, 40 important features are screened out through feature engineering. On this basis, Logistics regression model, Lasso-Logistics, Gradient Boosting Decision Tree (GBDT), Extreme Gradient Boosting (Xgboost), Light Gradient Boosting Machine (Lightgbm), and Gradient Boosting Categorical Features (Catboost) are established, and multiple learners are integrated. Finally, the constructed model is tested on data sets. The accuracy of the proposed model is 80.3%, the accuracy is 74.6%, the recall rate is 79.3%, and the running time is only 2.53 seconds. This means that the proposed model is superior to the previous models in terms of accuracy, precision, recall rate, and F1 value, and the time consumption is also in line with the actual engineering requirements. The proposed scheme provides some ideas for the research of machine learning technology in disease prediction.

## 1. Introduction

Gestational diabetes mellitus (GDM) is one of the major causes of type 2 diabetes and its syndromes spreading around the world. According to the research, by 2013, the number of people with GDM in China ranked second in the world. Machine learning algorithm focuses on studying the behavior rules and thinking patterns similar to human beings learned from massive knowledge, and reorganizes and processes the information to obtain new skills and optimization direction. Machine learning can combine relevant research contents in statistics, database, and knowledge graph to mine rules and iterate from massive data with sufficient computing resources [1]. Machine learning is becoming more and more mature and has been applied in many fields, especially in the fields of classification, clustering, and optimization, and has made great breakthroughs and wide applications in commercial scenarios such as search engines. In recent years, the application frequency and research depth of machine learning algorithm in the medical field grow rapidly. Some scholars have applied machine learning algorithm to predict the prevalence of some diseases, and achieved remarkable results. Ensemble learning is a special class of machine learning algorithms, which combines basic models based on the idea of integrating weak classifiers into strong classifiers, boosting the ability of model to prevent overfitting while ensuring accuracy. In addition to the stability and generalization ability of the integrated learning model compared with the traditional model, the final prediction accuracy is relatively high. At present, some integrated learning models are also applied in disease prediction, and the effect is remarkable. Therefore, using integrated learning algorithm to study the relationship between various indicators and GDM prediction model is one of the possible means to reduce the incidence, which is also worthy of study. GDM refers to the abnormal glucose metabolism of pregnant women during pregnancy. This type of diabetes is a temporary disease caused by pregnancy, but it will affect the safety of pregnant women and the fetus [2]. GDM patients are prone to high blood pressure, which is caused by insufficient insulin secretion and high blood sugar content in human body, thus affecting the elasticity of blood vessels. In addition, high blood sugar can promote the increase of amniotic fluid secreted by pregnant women, and stimulate the endometrium, which is prone to premature birth and suffocation. High blood sugar will also affect the immune system, affecting the phagocytosis of white blood cells, leading to a decline in immune capacity, and then the occurrence of placental abruption. Current studies have found that GDM is one of the causes of abnormal pregnancy, including fetal macrosomia and fetal shoulder dystocia. The influence of GDM goes beyond that. GDM will have long-term effects on the mother and fetus. Research results show that pregnant women with GDM have a 13%–63% probability of developing type 2 diabetes and abnormal glucose tolerance within five years after delivery. Therefore, the use of integrated algorithm to predict the incidence of GDM patients and constructing model interpretation of at-risk patients by improving model accuracy and existing data will contribute to the auxiliary diagnosis and prevention of GDM and contribute to intelligent diagnosis and reduction of adverse pregnancy, which is a worthy direction of in-depth research [3].

Gnanadass [4] pointed out that diabetes is the most common noninfectious disease in the world due to changes in dietary habits. The author used various machine learning algorithms to predict GDM and verified the accuracy of various machine algorithms with degree values. Deberneh and Kim [5] developed a machine learning model to predict the occurrence probability of type 2 diabetes in the next year using variables of the current year. The author used logistic regression, random forest, support vector machine, and integrated machine learning algorithm to predict the results. Hysing et al. [6] proposed that babies born at pregnancy-related risks face a series of developmental problems. This study was to investigate differences in sleep patterns between babies at pregnancy-related risk and those without these risk factors. Li et al. [7] pointed out that the important characteristics of diabetes explored by data mining analysis can be predicted and prevented. Based on this study, the author proposed a diabetes prediction algorithm based on Extreme Gradient Boosting (XGBoost) algorithm. The experimental results showed that the prediction accuracy of diabetes based on the improved feature combined with XGBoost algorithm was 80.2%, which was a feasible and effective method for diabetes prediction. Fitriyani et al. [8] proposed a disease prediction model based on individual risk factor data for early prediction of type 2 diabetes and hypertension. Many medical studies have been conducted on the factors of GDM, laying a foundation for data analysis of GDM. However, there is not a recognized most accurate index system and the most effective model, and there is still a lot of space to try and explore. Existing researches mostly use common regression methods, such as Logistics and a small amount of machine learning. Integrate algorithms can be used to predict GDM, hoping to improve the accuracy of model prediction.

Ensemble learning is a more characteristic category of machine learning algorithms, which combines basic models according to the idea of integrating weak classifiers into strong classifiers [9–11]. The ensemble learning model performs better in terms of stability and generalization ability relative to traditional models, and is relatively high in the final prediction accuracy. At present, some ensemble learning models are also utilized in disease prediction, and the effect is significant. Therefore, adopting the ensemble learning algorithm to study the relationship between various indicators and the GDM prediction model is one of the possible means to reduce the incidence of GDM, and it is also a topic worthy of research. GDM prediction model under cascade and ensemble learning algorithm is constructed by machine learning algorithm. The proposed model first performs feature selection through IV value analysis, which effectively removes redundant features and determines the final optimal feature subset to train the model. XGBoost, LightGBM (Light Gradient Boosting Machine), and Catboost (Gradient Boosting Categorical Features) models are adopted to build the GDM prediction model, and performance comparison was implemented to determine the model with optimal performance. Then, the idea of cascade is adopted to build the GDM prediction model with cascade structure and ensemble learning algorithm. The experimental results on the public data set show that the algorithm proposed can effectively reduce the possibility of overfitting of the model while improving the generalization ability and robustness of the model, which can achieve ideal prediction results. The main contribution of this work lies in the following aspects. The research perspective is relatively new. Most of the studies on GDM are based on the analysis of the risk factors affecting the pregnancy outcome of GDM, and few are based on the prediction of whether the pregnant woman is likely to develop GDM. This work focuses on the prediction of the risk of GDM. The application of research methods is innovative. Since most studies on GDM analysis use Logistics regression model, and few use machine learning method, let alone integrated learning method, to predict whether GDM has occurred, the integrated learning method is innovatively used in this work to establish the GDM prediction model and carry out the data prediction analysis.

## 2. Methodologies

Catboost [9–11] algorithm is an implementation of Boosting strategy in machine learning algorithm. Catboost and LightGBM [12–14] are similar to the XGBoost algorithm [15, 16], which both belong to the GBDT (Gradient Boosting Decision Tree) class of algorithms [17]. In contrast to LightGBM and XGBoost algorithms, the Catboost algorithm solves the problems that the previous algorithm cannot efficiently solve. It reasonably handles features, as well as the existence of gradient bias and prediction shift. To solve the above problems, Catboost mainly makes two improvements based on GBDT: processing the nominal attributes and solving the prediction offset to reduce the occurrence of overfitting.

### 2.1. GBDT Algorithm

GBDT is a kind of boosting algorithm, which can be regarded as an additive model composed of M trees. At each step of the GBDT algorithm, a decision tree is utilized to fit the residual of the current learner to obtain a new learner. After the decision tree of each step is combined, a strong learner is obtained [18]. GBDT algorithm model is shown in the following equation .

(1) $$\begin{array}{c} F\left(x,\omega \right)=\sum_{m=0}^{M}\alpha_{m}h_{m}\left(x,\omega \right)=\sum_{m=0}^{M}f_{m}\left(x,\omega_{m}\right). \end{array}$$

In equation (1), *x* is the input sample; *ω* is the model parameter; *h* is the classification regression tree; and *α* is the weight of the tree. The purpose of the algorithm is to obtain the final regression tree: *F*_*m*_.

The GBDT algorithm can be divided into 3 steps.

(I) First, a weak learner F_0_ (*X*) is initialized, as shown in the following equation.
  (2) $$\begin{array}{c} F_{0}\left(X\right)=\text{argmin}\sum_{i=1}^{N}L\left(y_{i},c\right). \end{array}$$
In equation (2), *y*_*i*_ is an element in the output space, *c* is the intermediate parameter of function derivation.
(II) M classification trees are established, the response value of each tree is calculated as shown in equation (3), and the best fit value is calculated as shown in equation (4).
  (a) Find the response value corresponding to each tree.
    (3) $$\begin{array}{c} r_{m,i}=-{\left[\frac{\partial L\left(y_{i}F\left(x_{i}\right)\right)}{\partial F\left(x\right)}\right]}_{F\left(x\right)=F_{m-1}\left(x\right)}. \end{array}$$
  In equation (3), *m* is the *m*th tree.
  (b) Fit the data using CART regression tree.
  (c) Calculate the best fit value.
    (4) $$\begin{array}{c} c_{m,j}=\text{argmin}\sum_{x_{i\in R_{m.j}}}L\left(y_{i},F_{m-1}\left(x_{i}\right)+c\right). \end{array}$$
  In equation (4), *F*_*m*−1_ is a strong learner.
  (d) Update the strong learner *F*_*m*_(*x*).
(III) The expression of the strong learner *F*_*M*_(*x*) is obtained.

(6) $$\begin{array}{c} F_{M}\left(x\right)=F_{0}\left(x\right)+\sum_{j=1,m=1}^{J_{m,c}}c_{m,j}I\left(x\in R_{m,j}\right). \end{array}$$

In equation (6), *F*_*M*_(*x*) is the final strong learner.

### 2.2. Catboost Algorithm

Catboost is the open-source machine learning library of Russian search giant Yandex in 2017. It is a member of the Boosting family of algorithms, and is also an improved implementation under the framework of GBDT algorithm. The main problem that the Catboost algorithm solves is how to efficiently and reasonably deal with the problems of categorical features, gradient bias, and prediction shift, thereby reducing the occurrence of overfitting and improving the accuracy and generalization ability [19–21].

Catboost has two major advantages. One is that it processes categorical features during the training process instead of processing categorical features in the feature preprocessing stage. Another is that when a tree structure is chosen, the algorithm for calculating leaf nodes can avoid overfitting [22–24].

## 3. Model Design

In GDM prediction, the use of machine learning algorithm analysis accounts for only a few. Some scholars mix the price-sensitive model with five kinds of traditional machine learning algorithms and choose a can predict model the GDM future risk the most feasible model. This model is usually added to many dangerous factors, Logistics, and other methods to the risk assessment of GDM. Then, the risk groups of GDM are identified according to the calculation results, or the risk factors are scored, and the risk groups are identified according to the scoring results. This model can effectively manage GDM, reduce the risk, and reduce the cost.

The research on GDM prediction includes the following aspects: data collection, data preprocessing, feature selection, model prediction, multimodel cascade, and result analysis, as shown in Figure 1.

Before model establishment and prediction, data need to be divided into training set and test set. Training set is used for model establishment, and test is used to verify whether the model is effective. The data has been divided in Section 3. The general prediction process is as follows. I. According to the principle of the algorithm, the data of the training set is used to establish the model and confirm the hyperparameters. II. The data of the test set is submitted into the trained model to predict the samples of the test set, and it is judged whether the samples suffer from GDM. III. The disease results predicted by the test set are compared with the real results to calculate the AUC (Accuracy), judge the quality of the model, and select an effective model.

### 3.1. Data Source

The data in this article comes from the data set commissioned by Beijing Qingwutong Health Technology Company published in the Tianchi Big Data Competition held by Alibaba. There are a total of 1000 training samples and 85-dimensional features in the data set. Among the 85-dimensional features, 30 are physical indicators, such as age, height, weight, BMI, and cholesterol indicators. The other 55 are genetic features. The values of 0, 1, and 2 in genetic features represent allelic genes AA, Aa, and aa in biology, respectively.

### 3.2. Data Preprocessing

Model training uses Graphic Processing Unit (GPU) server, hardware configuration is Intel E52665X2, 32 GRECC DDR3, 250G solid state disk, NVIDIA RTX 2080TI 11G graphics card 4. The software configuration is Ubuntu Linux 16.04, CUDA10.0, cuDNN7.6. The test is carried out on a laptop computer with Intel i79750H 4.5 GHz 6-core hardware, 32G DDR4 2666 memory, and GeForce GTX 1650 GPU. The software configuration is Windows10, CUDA10.1, Cudnn7.6, OpenCV3.4.1.

Medical data is characterized by containing many missing values and many outliers and meaningless values. The data processing in this work is mainly consisted of four steps. I. Since some data are with a missing ratio of more than 75%, it is difficult to fill in a reasonable method, and the weight of the impact on the prediction model is small. Therefore, these basic features with a high percentage of missing are determined to be eliminated. II. The basic features and outliers that have no effect on the prediction model are removed. III. The nearest neighbor imputation method is adopted for the data with a low percentage of missing data, and the missing data are imputed. IV. The one hot coding is performed for discrete variables SNP*∗*, BMI classification, and ACEID, respectively, as SNP1_1, SNP1_2, SNP1_3, SNP1_null, SNP2_1, SNP2_2, SNP2_3, SNP2_null, BMI classification_1, BMI classification_2, ACEID_1, and ACEID_2. With SNP1_3 as an example, SNP1 takes a value of 3 as a single feature.

### 3.3. Feature Selection

Feature selection plays a key role in modeling prediction at the later stage, especially in the case of small sample size and many features, noise elimination and correct feature selection will improve the accuracy and stability of the model. Based on the characteristics of small sample size and many missing values of the data set utilized in this work, as well as the interpretability of the feature analysis results, information value (IV) analysis and residual analysis are adopted to rank the importance of features, respectively.

IV value analysis measures the impact of a feature in the data on the target. The basic idea of IV value analysis is comparing the correlation degree by using the ratio of positive and negative samples occupied by a certain feature and the ratio of positive and negative samples in the overall data. The calculation is as follows.

(7) $$\begin{array}{c} p=\sum_{i}^{n}\left(P_{yi}-P_{ni}\right)*\text{ln}\frac{P_{yi}}{P_{ni}}. \end{array}$$

In equation (7), *n* is the number of variable groupings, *P*_*ni*_ is the proportion of positive samples contained in the *i*th group of data in the sample to the positive samples in all data, and *P*_*yi*_ is the proportion of negative samples contained in the *i*th group of data in the sample to the negative samples in all data. Taking VAR00007 feature as an example, the prevalence rate and IV value results of each feature value are calculated, as shown in Table 1.

From Table 1, after excluding of the Null value, the morbidity rate also increases with the increase of VAR00007. Especially, after the value of VAR00007 reaches 1.769, the morbidity rate almost reaches 0.8, which is a very high rate, indicating that this feature has a great influence on the morbidity.

Residual analysis is a univariate analysis method that can only provide first-order importance analysis. It is utilized to measure the relative degree of change in the ratio of positive and negative samples with the change in the value of a single variable. VAR00007 feature analysis is taken as an example to give the residual analysis results, as shown in Table 2.

Table 2 shows that the prevalence of VAR00007 is different in different groups or with different values, or the prevalence is gradually increasing or decreasing with the increase of value range.  Table 3 shows the eigenvalues.

Table 3 shows that VAR00007 contains the most information, followed by SNP37 features. SNP34 features contain slightly less information than SNP37, and Hypersensitive C-reactive protein and Pregnancy BMI features contain the least information.

The distribution of each variable is shown in Figures 2 and 3.

Figure 2 suggests that overweight and obese pregnant women are prone to have GDM.  Figure 3 reveals that the incidence rate is lower when SNP53 is missing. The reason may be that the SNP53 gene is not a gene that regulates the function of insulin and the secreted protein. IV value analysis method and residual error analysis method are utilized for feature selection, finally 9 feature variables that have an impact on diabetes are selected as input variables of the model, including age, pre-pregnancy BMI, hs-CRP, VAR00007, TG, RBP4, SNP53, SNP37, and SNP34. Among which, there are 6 continuous feature variables and 3 discrete feature variables.

### 3.4. Model Building

Three models are built in this work for GDM prediction, namely, XGBoost model, LightGBM model, and Catboost model. The model evaluation indicators are accuracy, recall rate, and F1 score. After data processing, cleaning, and feature selection, the data set is classified into training set and test set at a ratio of 7 : 3. The data are sent to different models for training separately, and a 7-fold cross-validation method is adopted for parameter tuning. The classification threshold affects the accuracy of the model. The method of dividing the threshold is utilizing the interval accuracy of the sample to determine the final threshold, the samples are sorted according to the predicted value, each 5% of which are divided and taken as an interval. Then, the interval where the accuracy of the last interval is greater than 50% is found, and the endpoint value of the interval is taken as the final threshold.

### 3.5. Selection of Evaluation Indicators

In this work, accuracy, precision, and recall rate are chosen to evaluate the model. Accuracy refers to the proportion of the number of samples with correct prediction to the total number of samples. Precision refers to the ratio of the number of samples predicted to be 1 and correctly predicted to the number of samples predicted to be 1. Recall rate refers to the ratio of the number of samples whose prediction is 1 and correctly predicted to the number of samples whose true value is 1. F1 value is the harmonic average of accuracy and recall rate. Precision, recall rate, and F1 value are chosen as evaluation indicators. Considering the engineering significance of the model, the calculation speed of the model also appears as an evaluation indicator.

(8) $$\begin{array}{c} P=\frac{TP}{TP+FP}. \end{array}$$

(9) $$\begin{array}{c} R=\frac{TP}{TP+FN}. \end{array}$$

(10) $$\begin{array}{c} F1=\frac{2PR}{P+R}. \end{array}$$

In equations (8) to (10), TP represents true positive, FP represents false positive, and FN represents false negative.

### 3.6. Multimodel Fusion Based on Cascade Classifier Method

To improve the performance of the model, the idea of cascading is utilized to improve the single model explained in the previous section. Before different models are cascading, the threshold input of cascading needs to be determined. Considering the actual meaning of the threshold, a conclusion can be drawn. Within a threshold range of any width, it is meaningful to predict the accuracy of samples falling within this threshold range greater than 50%. If the accuracy is not up to 50%, it has no practical significance.

From Figure 4, the ratio of positive and negative samples in the training set and test set adopted is about 1 : 1.1, so the cascade threshold is set to 0.5. The commonly used fusion methods of F1 models are mean method of regression prediction model and voting method of classification model, which are usually used for the fusion of weak classifiers. Because the constructed model is not a weak classifier model, these model fusion methods are not applicable. The evaluation index of the adopted data set is F1 value, so improving the model performance means improving the F1 value of the model, and improving the accuracy or recall rate of the model can also improve the F1 value of the model. Therefore, other classifiers are used to make a second judgment on the sample data whose threshold value is less than 0.5, so as to reduce the possibility of data being misclassified, improve the recall rate and accuracy of the model, and thus improve the F1 value of the model.

## 4. Analysis of Experimental Results

### 4.1. Model Test

The performances of the constructed XGBoost model, LightGBM model, and Catboost model on the test set are as shown in Figures 5 and 6.

From Figure 5, the accuracy of Catboost algorithm is 0.771, the accuracy is 0.700, the recall rate is 0.780, and the F1 value is 0.720. The accuracy of LightGBM algorithm is 0.725, the accuracy is 0.676, the recall rate is 0.673, and the F1 value is 0.674. The overall performance of Catboost and LightGBM is better than that of XGBoost.

GDM prediction performance is shown in Figure 5, and no matter which feature selection method is utilized for the training of the Catboost model, the Catboost model is superior to XGBoost model and the LightGBM model in terms of accuracy and precision. From the contrast of Figures 5 and 6, the accuracy and precision of the feature training model extracted using the IV value are higher relative to feature training model extracted using the residual method. Moreover, it is worth mentioning that due to the particularity of medical data, the recall rate is also an important reference factor in model evaluation. The recall of the proposed model is 1.07 percentage points higher versus that of the LightGBM model. The experimental results show that the Catboost model has strong superiority in processing the features of the data, and performs best on the issues raised.

### 4.2. Experimental Results and Analysis

Under the same conditions, the XGBoost model, the LightGBM model, and the Catboost model are utilized as models 1, 2, and 3 for the experiment, respectively. The experimental results are shown in Table 4.

After cascading, the F1 value of XGBoost model, LightGBM model, and Catboost model are all improved in contrast to the previous single model. When the Catboost model is utilized as the model 1, the F1 value of the cascade model is increased to 0.763 from 0.721 of single model, with an increase of 4.2%. When the LightGBM model is utilized as the model 1 and the Catboost model is utilized as the model 2, the F1 value of the cascade model is increased to 0.701 from 0.664 of single model, with an increase of 4.2%. When the XGBoost model is utilized as model 1 and the Catboost model is utilized as model 2, the F1 value of the cascaded model increases less. When the three sub-models are all Catboost models, the cascade model works best.

The model proposed in this work is compared with the model proposed by Jianyu Yu et al. On the same data set, the F1 value of the model proposed by Jianyu Yu et al. is 0.726, and the F1 value of model proposed in this work is 0.793, with an increase of 6.7%. The proposed model is compared with the Catboost single model on the same data set, and results show that the cascaded model has a significant increase in test time versus single model. However, when it comes to precision, accuracy, recall rate, and F1, the cascaded model is superior to Catboost single model, as shown in Table 5.

## 5. Conclusion

Against the background that GDM often has no obvious symptoms, which is easily missed, and delayed treatment is harmful to pregnant women and fetuses, the data set commissioned by Beijing Qingwutong Health Technology Company published in the Tianchi Big Data Competition held by Alibaba is taken as the experimental database. Then, GDM prediction model based on cascade and ensemble learning algorithm is built, to realize the early prediction of GDM. On the data set utilized in this work, the accuracy of the proposed prediction model is 80.3%, the precision is 74.6%, and the recall rate is 79.3%.

The proposed algorithm can provide effective guidance for GDM prediction, and has a very positive significance for protecting the health of pregnant women and fetuses. However, there are still some unfinished works in this article. For example, when the GDM prediction is performed, only the algorithms in machine learning are adopted. In the follow-up research, it will consider adopting the Long Short-Term Memory (LSTM) network in deep learning for GDM prediction. In conclusion, the proposed model has favorable adoption value in GDM prediction.

## Figures and Tables

**Figure 1:** GDM prediction model.

**Figure 2:** BMI before pregnancy and average prevalence.

**Figure 3:** SNP53 value and average prevalence.

**Figure 4:** Classifier structure diagram.

**Figure 5:** Comparison of evaluation indicators of XGBoost model, LightGBM model, and Catboost single model (residual analysis).

**Figure 6:** Comparison of evaluation indicators of XGBoost model, LightGBM model, and Catboost single model (IV value analysis).

**Table 1:** IV analysis results of some data.

Column name	Characteristic values	The total number of	Prevalence rate (%)	Relative prevalence	Item IV	Total IV
VAR00007	[1.20, 1.48)	166	24.3	−48.5%	15.60	67.16
VAR00007	[1.44, 1.52)	177	33.5	−28.3%	5.59	67.16
VAR00007	[1.46, 1.53)	185	39.6	−15.7%	1.75	67.16
VAR00007	[1.52, 1.63)	224	45.7	−2.8%	0.071	67.16
VAR00007	≥1.60	238	79.2	69.6%	44.47	67.16
VAR00007	Null	10	70.1	49.3%	0.89	67.16

**Table 2:** Residual analysis results of some data.

Field meaning	Sequence	Value	Number of people	Prevalence rate (%)	Relative prevalence
VAR00007	36	B [1.20, 1.48)	256	27.2	−19.7%
VAR00007	36	C [1.44, 1.52)	272	37.3	−9.4%
VAR00007	36	D_[1.46, 1.53)	222	45.6	−1.4%
VAR00007	36	E_[1.52, +Inf)	240	78.9	−32.8%
VAR00007	36	Missing value	10	70.1	24.1%

**Table 3:** Variable names, types, and IV values selected in this work.

Variable name	IV value	Variable types
Age	0.17	Continuous variables

Pregnancy BMI	0.12	Continuous variables

Hypersensitive C-reactive protein	0.12	Continuous variables

VAR00007	0.37	Continuous variables

Triglycerides	0.15	Continuous variables

RBP4	0.16	Continuous variables

SNP53	0.17	Discrete variable
SNP37	0.34	Discrete variable
SNP34	0.33	Discrete variable

**Table 4:** Comparison of cascade results of models.

Model no. 1	Model no. 2	Model no.3	F1	Ascension degree (%)
Catboost	XGBoost	Catboost	0.732	1.1%
	LightGBM		0.741	2%
	Catboost		0.763	4.2%

Catboost			0.721	—
LightGBM	XGBoost	Catboost	0.683	1.9%
	LightGBM		0.692	2.8%
	Catboost		0.701	3.7%

LightGBM			0.664	—
XGBoost	XGBoost	Catboost	0.673	0.5%
	LightGBM		0.682	0.4%
	Catboost		0.691	1.3%

XGBoost			0.678	

**Table 5:** Comparison of parameters of models.

Model	Accuracy	Precision	Recall	F1	Time
Cascade model proposed	0.803	0.746	0.821	0.793	2.53
Model proposed by Yu et al. [25]	—	—	—	0.726	—
Catboost single model	0.783	0.726	0.781	0.721	0.932

## Data Availability

The data used to support the findings of this study are included within the article.
